The article "Value of CT Radiomics and Clinical Features in Predicting Bone Metastases in Patients with NSCLC" was retracted in 2023. Reasons: signs of a paper mill; suspected computer-generated content; unreliable results or conclusions; lack of ethics approval or compliance.

# Value of CT Radiomics and Clinical Features in Predicting Bone Metastases in Patients with NSCLC

**DOI:** 10.1155/2022/7642511

**Published:** 2022-08-22

**Authors:** Lu Chen, Lijuan Yu, Xueyan Li, Zhanyu Tian, Xiuyan Lin

**Affiliations:** ^1^Hainan Cancer Hospital (Affiliated Cancer Hospital of Hainan Medical College), Nuclear Medicine Department, Haikou, China; ^2^College of Bioinformatics, Hainan Medical University, Haikou, China

## Abstract

**Objective:**

To explore the CT radiomic features and clinical imaging features of the primary tumor in patients with nonsmall cell lung cancer (NSCLC) before treatment and their predictive value for the occurrence of bone metastases.

**Methods:**

From June 2017 to June 2021, 195 patients with NSCLC who were pathologically diagnosed without any treatment in the Cancer Hospital Affiliated to Hainan Medical College were retrospectively analyzed, and they were divided into a bone metastasis group and a nonbone metastasis group. The relationship between clinical imaging features and bone metastasis in patients was analyzed by the *t*-test, rank sum test, and *χ*^2^ test. At the same time, ITK software was used to extract the radiomic characteristics of the primary tumor of the patients, and the patients were randomly divided into a training group and a validation group in a ratio of 7 : 3. The training model was validated in the validation group, and the performance of the model for predicting bone metastases in NSCLC patients was verified by the ROC curve, and a multivariate logistic regression prediction model was established based on the omics parameters extracted from the best prediction model combined with clinical image features.

**Results:**

Seven features were screened from the primary tumor by LASSO to establish a model for predicting metastasis. The area under the curve was 0.82 and 0.73 in the training and validation sets. The best omics signature and univariate analysis suggested clinical imaging factors (*P* < 0.05) associated with bone metastases were included in multivariate binary logistic analysis to obtain clinical characteristics of the primary tumor such as gender (OR = 0.141, 95% CI: 0.022–0.919, *P* = 0.04), increased Cyfra21-1 (OR = 0.12, 95% CI: 0.018–0.782, *P* = 0.027), Fe content in blood (OR = 0.774, 95% CI: 0.626–0.958, *P* = 0.018), CT signs such as lesion homogeneity (OR = 0.052, 95% CI: 0.006–0.419, *P* = 0.006), pleural indentation sign (OR = 0.007, 95% CI: 0.001–0.696, *P* = 0.034), and omics characteristics glszm_Small Area High Gray Level Emphasis (OR = 0.016, 95% CI: 0.001–0.286, *P* = 0.005) were independent risk factors for bone metastasis in patients.

**Conclusion:**

The prediction model established based on radiomics and clinical imaging features has high predictive performance for the occurrence of bone metastasis in NSCLC patients.

## 1. Introduction

Lung cancer is the malignant tumor with the highest incidence in the world. Among them, nonsmall cell lung cancer (NSCLC) is very easy to metastasize through the blood system, and bone metastasis is a common distant metastasis of lung cancer, with an incidence of about 50% [1], where bone metastases often predict shortened patient survival and decreased quality of life. The median survival time after bone metastases in lung cancer patients is only 6–10 months, and 46% of lung cancer patients with bone metastases are complicated by skeletal-related events (SREs) [2], such as hypercalcemia, pathological fractures, spinal cord compression, and other complications that seriously affect the quality of life of patients [3]. For patients with bone metastases, the current treatment standard includes palliative radiotherapy such as external beam radiotherapy. However, the local control rate of patients is low [4–6]. Therefore, exploring new treatment methods for bone metastasis is of great significance to improving the quality of life of patients.

Since Lambin et al. [7] proposed the concept of radiomics in 2012, it has developed rapidly by extracting quantitative features of lesions through high-throughput images to describe tumor phenotype and heterogeneity from a macroscopic perspective. A large number of studies have also focused on the relationship between radiomics and lymph node metastasis and brain metastasis [8–10], including metastasis of NSCLC [11]. In view of this, this study aimed to apply the method of radiomics to explore the CT radiomic characteristics and clinical characteristics of NSCLC patients and their predictive value for the occurrence of bone metastases.

In view of the above research basis, at present, the relationship between clinical imaging features and bone metastasis in patients was analyzed by *t*-test, rank sum test, and *χ*2 test. At the same time, ITK software was used to extract the radiomic characteristics of the primary tumor of the patients, and the patients were randomly divided into the training group and the validation group in a ratio of 7 : 3. The training model was validated in the validation group, and the performance of the model for predicting bone metastases in NSCLC patients was verified by the ROC curve, and a multivariate logistic regression prediction model was established based on the omics parameters extracted from the best prediction model combined with clinical image features.

## 2. Data and Methods

### 2.1. Objects

From June 2017 to June 2021, the clinical and imaging data of 501 newly diagnosed lung cancer patients admitted to the Cancer Hospital Affiliated to Hainan Medical College were retrospectively analyzed. The diagnostic criteria for bone metastases [12–14]areas follows: (1) whole body SPECT/CT bone scan prompts, if there are metastatic lesions, the positive judgment criteria refer to the diagnostic criteria for bone metastases in the literature, and all bone imaging results are jointly diagnosed by more than 2 physicians. The termination time for judging the presence of bone metastases in the patient is December 31, 2021, or the patient's death; (2) puncture biopsy. Inclusion criteria were as follows: (1) all patients had a clear pathological diagnosis, and the pathological type was nonsmall cell lung cancer; (2) the first visit, without surgery, chemotherapy, or radiotherapy; (3) all patients underwent chest CT examination or PET/CT examination within 7 days of visit; (4) no history of other malignancies. Exclusion criteria were as follows: (1) CT images with heavy motion artifacts or unclear boundary between tumor and surrounding tissue, unable to accurately delineate the boundary; (2) patients with incomplete information. Finally, 195 patients were included.

### 2.2. Basic Information

The collected information includes the basic clinical information of patients such as gender, age, smoking history, family history, pathological type, blood iron (Fe), hemoglobin, alkaline phosphatase (ALP), blood calcium concentration, serum CEA, CA125, Cyfra21-1, NSE, etc., imaging characteristics of primary tumor lesions, regional lymph node metastasis, and other distant metastasis.

### 2.3. Data Processing and Model Building

The volume of interest (VOI) of the tumor was delineated layer by layer by ITK software, and the file was imported into Python. Before analysis, the data were excluded from missing values and standardized. Then, the data set was randomly divided into the training group and the validation group with a ratio of 7 : 3 by the random grouping method. Univariate correlation analysis and the LASSO (least absolute shrinkage and selection operator logistic regression, LLR) regression model were used to select CT features. After 5-fold cross-validation, the omics features were selected and included in the support vector machine (SVM) model according to the least square error criterion machine model, and the predictive ability was judged by the area under the curve (AUC) of the receiver operating characteristic (ROC).

By using SPSS 25.0 statistical software, using *t*-test, Mann-Whitney *U* test, and *χ*^2^ test analysis, clinical imaging indicators (*P* < 0.05) and omics characteristics were included in multivariate binary logistic regression analysis to find independent risk factors for bone metastases in patients with NSCLC.

## 3. Results

### 3.1. Clinical Imaging Characteristics and Univariate Analysis of All the Patient Count Data

A total of 195 patients, aged 34–93 years, were included in this study, with an average of 60.56 ± 10.114 years. There were 144 patients with bone metastases from lung cancer, with an average age of 60.67 ± 10.605 years. There were 51 patients without bone metastases, with an average age of 60.25 ± 8.667 years. For details, see Tables 1 and 2.

### 3.2. Clinical Imaging Features and Univariate Analysis of Measurement Data of All Patients

The clinical and imaging measurement data and univariate analysis results (see Table 3) with statistically significant measurement data were subjected to ROC curve analysis, and the Youden index was used to determine the diagnostic boundary value. The results showed that the diagnostic boundary values of ALP, Fe, and the shortest diameter of the largest lymph node were 69.5 mmol/L, 10.65 ng/ml, and 6.5 mm, respectively (Table 4, Figure 1).

### 3.3. CT Radiomics Model Establishment and Univariate Analysis

The alpha value of LLR = 0.0160 (Figure 2), the SVM training set score is 0.74, and the test set score is 0.75. Based on the established training set data, the 7 best CT omics features are finally retained. The distribution of some image features is shown in Figure 3. In order to test the predictive performance of the radiomics label for bone metastases in patients, we used the ROC curve to analyze its predictive results and judged its predictive ability according to the sizes of the area under the curve (AUC) (Figure 4) which are 0.73 and 0.82.

Substituting CT omics parameters into binary Logistic regression analysis results showed that shape_Sphericity, glcm_Imc1, and glszm_ Small Area High Gray Level Emphasis among CT omics parameters had statistical significance on bone metastasis in NSCLC patients (*P* < 0.05), while other characteristic parameters had no significant effect on bone metastasis (*P* > 0.05) (Table 5).

### 3.4. Multifactor Analysis

The clinical characteristics of risk factors identified in univariate analysis (sex, pathological type, serum CEA, NSE, Cyfra21-1, and ProGRP levels were increased), CT signs (lesion density, lesion homogeneity, burr sign, pleural depression sign, pleural effusion and lymph node, and lung, brain, adrenal, or other site metastasis), and CT omics characteristic parameters (shape_Sphericity, glcm_Imc1, and glszm_SmallAreaHighGrayLevelEmphasis) were included in the multivariate binary logistic regression equation for multivariate analysis, to further explore the impact of NSCLC Independent risk factors for bone metastases in patients (see Table 6). It can be known from the table that the clinical characteristics of patients such as gender (OR = 0.141, 95% CI: 0.022–0.919, *P* = 0.04), increased Cyfra21-1 (OR = 0.12, 95% CI: 0.018–0.782, *P* = 0.027), Fe content in blood (OR = 0.774, 95% CI: 0.626–0.958, *P* = 0.018), CT signs such as lesion homogeneity (OR = 0.052, 95% CI: 0.006–0.419, *P* = 0.006), pleural indentation sign (OR = 0.007, 95% CI: 0.001–0.696, *P* = 0.034), and the omics feature glszm_SmallAreaHighGrayLevelEmphasis (OR = 0.016, 95% CI: 0.001–0.286, *P* = 0.005) were associated with bone metastases from lung cancer independent risk factors.

## 4. Discussion

Bone metastasis is a common cause of death in lung cancer patients, which seriously affects the quality of life and survival of NSCLC patients [15, 16]. How to effectively predict bone metastasis from lung cancer and reduce the incidence is the most concerned issue of thoracic surgeons and lung cancer patients [17]. In this study, we believe that patients with bone metastases may have special clinical imaging features and radiomic characteristics that can be differentiated from patients with nonbone metastases. By analyzing and studying these variables, a predictive model for bone metastases from lung cancer can be established and can guide clinical diagnosis and treatment according to the prediction model.

In this study, various clinical and imaging characteristics of NSCLC patients were statistically analyzed. The results showed that gender was an influencing factor in the occurrence of bone metastases from lung cancer. Male patients were more likely to develop bone metastases than female patients. It is consistent with the conclusion that gender is a high-risk factor for bone metastasis, and some studies suggest that it may be related to the protective effect of estrogen [16, 17]. As a nonorgan-specific tumor marker, Cyfra21-1 is not affected by lung diseases such as pneumonia and bronchus, as well as age, gender, and other factors, but it is significantly expressed in lung cancer patients [18]. Zhang et al. [19] and other studies showed that Cyfra21-1 is more important than neuron-specific enolase (NSE) and carcinoembryonic antigen (CEA) in the occurrence and prognosis of lung cancer metastasis. In this study, the level of Cyfra21-1 in the bone metastasis group was higher than that in the nonbone metastasis group, and the difference was statistically significant. Early investigators demonstrated that dysregulation of iron-regulated pathways and the concomitant accumulation of excess iron promote tumor growth [20]. The low expression of ferroportin (FPN) in NSCLC can lead to enhanced migration and proliferation of lung cancer cells and the accumulation of intracellular iron ions, thereby forming a migration and carcinogenic effect [21]. Whether NSCLC has distant metastasis was significantly correlated. The results of this study suggest that the risk of bone metastases in patients with high serum Fe content is higher than that in normal patients. In this study, the specificity of 10.65 ng/ml for the diagnosis of bone metastases in NSCLC was 83.3% [22]. Whether the density of primary lesions is uniform also reflects the difference in the growth and proliferation rate of malignant tumor cells and tumor burden to some extent. When the tumor shows partial liquefaction and necrosis, it indicates that the tumor is overloaded, and the metastatic potential is closely related to the tumor burden [23]. The pleural depression sign is caused by the scar tissue in the tumor pulling the adjacent visceral pleura. In the scar tissue of the tumor, there are changes in arachidonic acid metabolism, the overexpression of eicosanoid signaling genes, and the remodeling of alveolar capillaries, which are conducive to the shedding of tumor cells, indicating that the tumor foci with CT signs of pleural depression have great potential for distant metastasis [24]. Glszm_SmallAreaHighGrayLevelEmphasis is a small area of high gray emphasis in the gray area size matrix and is a texture feature. The larger the value, the greater the texture heterogeneity in the area [25]. Studies have shown that Glszm-related features are associated with aggressiveness, and highly aggressive lung cancer patients are more prone to bone metastases [26].

The clinical treatment of bone metastases from lung cancer is relatively passive. Most patients are in the terminal stage of the disease when they are discovered. Traditional methods lack a complete scoring system. By analyzing the characteristics of bone metastases from lung cancer and building a corresponding prediction model, it can help doctors predict the possibility of bone metastases in lung cancer patients more quickly and accurately, which is very important to guide clinical decision-making, but relevant research and reports are still limited. In this study, after analyzing the clinical imaging and omics characteristics of patients with bone metastases from lung cancer, an omics prediction model was built, the relevant independent risk factors were extracted, and corrected by multivariate regression analysis. The model was considered to have a good prediction ability to help clinicians differentiate and assess the risk of skeletal involvement and to specifically recommend closer investigations in patients without distant metastases. In addition, we can use this model variable to distinguish the prognosis of patients with bone metastases, so as to achieve more precise treatment for lung cancer patients. This study also has limitations. First, as a retrospective study, our proposed hypothesis requires larger data volumes and advanced follow-up modalities for follow-up. Secondly, this study adopts a single-center retrospective study, which lacks external data for verification. If further multicenter prospective studies can be conducted, they will have more clinical value.

In conclusion, this study used noninvasive examination of patients as an influencing factor to construct a prediction model and realized the prediction of bone metastases from lung cancer. This model is helpful for the clinical individualized treatment of lung cancer patients.

## Figures and Tables

**Figure 1:** ROC curves of ALP (a), Fe (b), and maximum short diameter of the lymph nodes (c) in predicting osseous metastasis for NSCLC patients.

**Figure 2:** LASSO-logistic regression screening for the radiomic characteristics of NSCLC patients with bone metastasis. (a) Convergence graph of 51 radiomic feature coefficients, the horizontal axis is log lambda, and the vertical axis is the radiomic feature weighting coefficient; (b) cross-validation graph, the horizontal axis is log(lambda). The vertical axis is MSE. Different lambda values correspond to different MSEs. The vertical dotted line in the figure represents the number of optimal radiomic features selected by LASSO regression using 5-fold cross-validation. According to the minimum MSE criterion, when *λ* = 0.0160, the optimal model is obtained; (c) finally, 7 radiomic features were selected.

**Figure 3:** Distribution map of imaging omics characteristics affecting bone metastasis in NSCLC patients screened by the Lasso-logistic regression.

**Figure 4:** ROC curves for osseous metastasis using radiomics signature. (a) ROC curve for predicting osseous metastasis using radiomics signature in the train group. (b) ROC curve for predicting osseous metastasis using radiomics signature in the validation group.

**Table 1:** Patients' characteristics and detailed information.

Characteristics		Osseous metastasis (*N* = 144)	No osseous metastasis (*N* = 51)	*χ * ^2^	*P* value
Gender, *n* (%)	Male	104 (53.3%)	28 (14.4%)	5.166	0.023*∗*
	Female	40 (20.5%)	23 (11.8%)		

Age/year, *n* (%)	30–45	9 (4.6%)	1 (0.5%)	2.532	0.47
	45–60	56 (28.6%)	25 (12.8%)		
	60–75	67 (34.4%)	21 (10.8%)		
	＞75	12 (6.2%)	4 (2.1%)		

Histology	Squamous carcinoma	14 (7.2%)	12 (6.2%)	7.055	0.029*∗*
	Adenocarcinoma	127 (65.1%)	39 (20%)		
	Not classified	3 (1.5%)	—		

Smoking history	Yes	48 (24.6%)	18 (9.2%)	0.065	0.799
	No	96 (49.2%)	33 (16.9%)		

Family history	Yes	7 (3.6%)	3 (1.5%)	0.081	0.776
	No	137 (70.3%)	48 (24.6)		

Blood calcium	Reduce level 1	28 (14.4%)	4 (2.1%)	5.777	0.123
	Reduce level 2	9 (4.6%)	2 (1.0%)		
	Reduce level 3	3 (1.5%)	—		
	Normal	104 (53.3%)	45 (23.1%)		

Blood CEA	1	105 (53.8%)	9 (4.6%)	47.375	0.001*∗*
	0	39 (20.0%)	42 (21.5%)		

Blood NSE	1	64 (32.8%)	11 (5.6%)	8.327	0.004*∗*
	0	80 (41.0%)	40 (20.5%)		

Blood Cyfra21-1	1	107 (54.9%)	18 (9.2%)	24.908	0.001*∗*
	0	37 (19.0%)	33 (16.9%)		

Blood ProGRP	1	42 (21.5%)	2 (1.0%)	13.737	0.001*∗*
	0	102 (52.3%)	49 (25.1%)		

Blood SCC	1	39 (20.0%)	11 (5.6%)	0.601	0.438
	0	105 (53.8%)	40 (20.5%)		

**Table 2:** Patients' primary image characteristics and detailed information.

Characteristics		Osseous metastasis (*N* = 144)	No osseous metastasis (*N* = 51)	*χ* ^2^	*P* value
Focal site	Superior lobe of right	42 (21.5%)	12 (6.2%)	2.596	0.870
	Middle lobe of right	7 (3.6%)	3 (1.5%)		
	Inferior lobe of right	32 (16.4%)	10 (5.1%)		
	Hilum of right	5 (2.6%)	2 (1.0%)		
	Superior lobe of left	33 (16.9%)	15 (7.7%)		
	Inferior lobe of left	23 (11.8%)	7 (3.6%)		
	Hilum of left	2 (1.0%)	2 (1.0%)		

Bronchial stenosis	1	72 (36.9%)	21 (10.8%)	1.175	0.278
	0	72 (36.9%)	30 (15.4%)		

Density	No glass	142 (72.8%)	39 (20%)	27.704	0.001*∗*
	Glass	2 (1.0%)	12 (6.2%)		

Uniform	No	116 (59.5%)	28 (14.4%)	7.934	0.005*∗*
	Yes	28 (14.4%)	20 (10.3%)		

Cavity	1	6 (3.1%)	3 (1.5%)	0.252	0.616
	0	138 (70.8%)	48 (24.6%)		

Calcification	1	8 (4.1%)	2 (1.0%)	0.207	0.649
	0	136 (69.7%)	49 (25.1%)		

Vein	1	143 (73.3%)	47 (24.1%)	7.704	0.006*∗*
	0	1 (0.5%)	4 (2.1%)		

Pleural depression	1	142 (72.7%)	42 (21.6%)	18.556	0.001*∗*
	0	2 (1.0%)	9 (4.6%)		

Leaflet	1	136 (69.7%)	45 (23.1%)	2.179	0.140
	0	8 (4.1%)	6 (3.1%)		

Obstructive pneumonia	1	17 (8.8%)	7 (3.6%)	0.117	0.732
	0	126 (64.9%)	44 (22.7%)		

Obstructive atelectasis	1	6 (3.1%)	5 (2.6%)	2.248	0.134
	0	138 (70.8%)	46 (23.6%)		

Pleural effusion	1	52 (26.7%)	8 (4.1%)	7.376	0.007*∗*
	0	92 (47.2%)	43 (22.1%)		

Pericardial effusion	1	21 (10.8%)	2 (1.0%)	4.115	0.43
	0	123 (63.1%)	49 (25.1%)		

Lymphatic metastasis	1	108 (55.4%)	23 (11.8%)	15.273	0.001*∗*
	0	36 (18.5%)	28 (14.4%)		

Intrapulmonary metastasis	1	42 (21.5%)	—	18.958	0.001*∗*
	0	102 (52.3%)	51 (26.2%)		

Pleural metastasis	1	10 (5.1%)	—	3.733	0.053
	0	134 (68.7%)	51 (26.2%)		

Brain metastases	1	55 (28.2%)	—	27.132	0.001*∗*
	0	89 (45.6%)	51 (26.2%)		

Adrenal metastasis	1	15 (7.7%)	—	5.798	0.016*∗*
	0	128 (66.0%)	51 (26.2%)		

Other organ metastases	1	17 (8.7%)	—	6.596	0.010*∗*
	0	127 (65.1%)	51 (26.2%)		

**Table 3:** Patients' categorical data characteristics and detailed information.

Characteristics	Osseous metastasis (*N* = 144)	No osseous metastasis (*N* = 51)	*P* value
Hemoglobin	124.37 ± 18.472	121.51 ± 15.369	0.321
ALK	146.17 ± 199.360	80.80 ± 51.939	0.001*∗*
Fe	8.362 ± 4.1867	11.894 ± 5.7049	0.001*∗*
The maximum long diameter	36.90 ± 21.608	34.88 ± 24.119	0.886
The maximum transverse diameter	27.09 ± 15.092	27.47 ± 19.581	0.279
Maximum short diameter of the lymph nodes	13.58 ± 7.592	9.71 ± 7.162	0.003*∗*

**Table 4:** The Yoden index determines the diagnostic limits for categorical data.

Characteristics	Sensitivity (%)	Specificity (%)	Diagnostic threshold	AUC
ALP	88.2	51	69.5 mmol/L	0.750
Fe	54.9	83.3	10.65 ng/ml	0.714
Maximum short diameter of the lymph nodes	87.5	51	6.5 mm	0.709

**Table 5:** Univariate binary logistic regression to determine the risk factors for bone metastasis.

Characteristics	*P*	OR	OR (95% CI)
shape_Flatness	0.771	0.660	0.040–10.802
shape_MajorAxisLength	0.275	1.016	0.988–1.044
shape_Sphericity	0.011^*∗*^	0.001	0.000–0.173
glcm_Imc1	0.017^*∗*^	5.689 E+11	196.845–1.6444 E + 18
glrlm_GrayLevelNonUniformityNormalized	0.801	2.084	0.007–635.485
glszm_SizeZoneNonUniformity	0.077	0.842	0.695–1.019
glszm_SmallAreaHighGrayLevelEmphasis	0.023^*∗*^	0.232	0.066–0.814

**Table 6:** Multivariate binary logistic regression to determine the independence risk factors for bone metastasis.

Characteristics	*P*	OR	OR (95% CI)
shape_Sphericity	0.271	0.004	0.001–80.597
glcm_Imc1	0.057	2.125E + 16	0.259–1.745 E + 39
glszm_SmallAreaHighGrayLevelEmphasis	0.005^*∗*^	0.016	0.001–0.286
ALP	0.329	1.009	0.991–1.028
Fe	0.018^*∗*^	0.774	0.626–0.958
Maximum short diameter of the lymph nodes	0.427	0.943	0.816–1.090
Gender	0.040^*∗*^	0.141	0.022–0.919
Histology	0.414	0.747	0.219–2.544
Blood CEA	0.781	0.753	0.102–5.572
Blood NSE	0.938	1.069	0.200–5.727
Blood Cyfra21-1	0.027^*∗*^	0.120	0.018–0.782
Blood ProGRP	0.973	1.044	0.084–12.910
Density	0.396	0.271	0.013–5.522
Uniform	0.006^*∗*^	0.052	0.006–0.419
Vein	0.739	2.211	0.021–233.082
Pleural depression	0.034^*∗*^	0.007	0.001–0.696
Pleural effusion	0.520	1.834	0.290–11.609
Lymphatic metastasis	0.143	0.184	0.019–1.770
Intrapulmonary metastasis	0.996	0.000	0.000–0.000
Brain metastases	0.994	0.000	0.000–0.000
Adrenal metastasis	0.999	0.000	0.000–0.000
Other organ metastases	0.998	0.000	0.000–0.000

## Data Availability

The datasets used and analyzed during the current study are available from the corresponding author upon reasonable request.
